The article "Effect of Rehabilitation Nursing under the Guidance of the Health Action Process Approach Model on Perioperative Nursing Effect of Artificial Hip Arthroplasty: Effect on Promoting Quality of Life and Postoperative Rehabilitation" was retracted in 2023. Reasons: unreliable results or conclusions; concerns about the data; concerns about the peer review; concerns about the citations.

# Effect of Rehabilitation Nursing under the Guidance of the Health Action Process Approach Model on Perioperative Nursing Effect of Artificial Hip Arthroplasty: Effect on Promoting Quality of Life and Postoperative Rehabilitation

**DOI:** 10.1155/2022/1247002

**Published:** 2022-04-12

**Authors:** Xiangfeng Meng, Yibing Yu

**Affiliations:** ^1^Department of Orthopaedic Surgery, The Fourth Hospital of Wuhan, Wuhan, 430030 Hubei Province, China; ^2^Department of Rehabilitation, The Fourth Hospital of Wuhan, Wuhan, 430030 Hubei Province, China

## Abstract

**Objective:**

To explore the influence of rehabilitation nursing under the guidance of Health Action Process Approach (HAPA) model on the perioperative nursing effect of artificial hip replacement and to analyze the effect of this nursing model on the quality of life and postoperative rehabilitation of patients undergoing artificial hip replacement.

**Methods:**

A total of 200 patients with hip arthroplasty treated in our hospital from January 2019 to July 2021 were enrolled. The patients were randomly assigned into the control group and study group. The former received routine nursing, and the latter received rehabilitation nursing under the guidance of the HAPA model. Nursing satisfaction, pain score, Harris hip function score, timed stand-up-walk test, MBI score, and quality of life score were compared.

**Results:**

First of all, we compared the nursing satisfaction. In the study group, 86 cases were very satisfied, 8 cases were satisfied, and 6 cases were general; the satisfaction rate was 100%. In the control group, 48 cases were very satisfied, 22 cases were satisfied, 12 cases were general, and 18 cases were dissatisfied; the satisfaction rate was 82.0%. The nursing satisfaction in the study group was higher compared to that in the control group (*P* < 0.05). Secondly, we compared the pain scores. Before nursing, there exhibited no significant difference (*P* > 0.05). After nursing, the pain score of the two groups increased. Moreover, the pain score of the study group at discharge and 1 month, 3 months, and 6 months after operation was lower compared to that of the control group (*P* < 0.05). Before nursing, there exhibited no significant difference in the Harris hip joint function score (*P* > 0.05). After nursing, the Harris hip function score increased. Furthermore, the Harris hip function score of the study group at discharge and 1 month, 3 months, and 6 months after operation was higher compared to that of the control group (*P* < 0.05). In terms of the timed stand-up-walking test, there exhibited no significant difference before nursing (*P* > 0.05). After nursing, the time of the timed stand-up-walk test in both groups decreased. And the timed stand-up-walk test at discharge and 1 month, 3 months, and 6 months after operation in the study group was lower compared to that in the control group (*P* < 0.05). Compared with the MBI scores, there exhibited no significant difference before nursing (*P* > 0.05). After nursing, the MBI scores increased. Of note, the MBI scores of the study group at discharge and 1 month, 3 months, and 6 months after operation were higher compared to those of the control group (*P* < 0.05). Finally, we compared the scores of life quality. Before nursing, there exhibited no significant difference (*P* > 0.05). After nursing, the scores of life quality decreased. The scores of physiological function, psychological function, social function, and health self-cognition in the study group were lower compared to those in the control group (*P* < 0.05).

The article "Effect of Rehabilitation Nursing under the Guidance of the Health Action Process Approach Model on Perioperative Nursing Effect of Artificial Hip Arthroplasty: Effect on Promoting Quality of Life and Postoperative Rehabilitation" was retracted in 2023. Reasons: unreliable results or conclusions; concerns about the data; concerns about the peer review; concerns about the citations.

**Conclusion:**

The perioperative rehabilitation nursing program of artificial hip replacement for the elderly based on the HAPA model is feasible, which can effectively enhance the functional recovery of hip joint, promote the ability of self-care of daily life, relieve pain and anxiety, and help to achieve dynamic balance and gait stability in the early stage. The rehabilitation program is better than routine nursing. As a new social cognitive model, the HAPA model is applied to the rehabilitation nursing environment of hip replacement from the aspect of social cognitive behavior, which can help to enhance the rehabilitation behavior of elderly patients, playing an important role in the rehabilitation effect of perioperative nursing.

## 1. Introduction

Hip fractures include femoral neck fracture (FNF), femoral intertrochanteric fracture (ITF), and femoral subtrochanteric fracture (SFF) [1]. Elderly hip fracture is known as “the last fracture in life” [2]. FNF means that the fracture site is located between the lower part of the femoral head and the base of the femoral neck, accounting for about 3.58% of body fractures and 53% of proximal femoral fractures [3]. ITF refers to fractures above the level of the lesser trochanter to the base of the femoral neck, accounting for about 3% of systemic fracture diseases and 35.7% of hip fractures [4, 5]. It is estimated that the number of elderly hip fractures will reach 2.6 million by 2025, and the number of elderly hip fractures will increase to 4.5 million by 2050 [6]. Most of the elderly hip fractures are low-energy injury, which has the characteristics of high fatality rate, high disability rate, many complications, high failure rate, and heavy burden [7]. Due to the poor body conditions and many basic diseases in elderly patients, most of them are accompanied by osteoporosis, anemia, hypoproteinemia, hypertension, diabetes, and other internal diseases, which may aggravate or complicate the original basic diseases after fracture [8]. In addition, the risk of surgical anesthesia in elderly patients is high, which brings many challenges for fracture surgery. Therefore, early surgery, early sitting up, or early getting out of bed is the most important way to reduce complications and mortality, which can bring a good prognosis.

The article "Effect of Rehabilitation Nursing under the Guidance of the Health Action Process Approach Model on Perioperative Nursing Effect of Artificial Hip Arthroplasty: Effect on Promoting Quality of Life and Postoperative Rehabilitation" was retracted in 2023. Reasons: unreliable results or conclusions; concerns about the data; concerns about the peer review; concerns about the citations.

There are a variety of surgical treatments for hip fracture in the elderly, mainly internal fixation and artificial hip arthroplasty [9]. FNFs are often treated with artificial hip replacement, intertrochanteric fractures can be treated with artificial hip replacement or fixation, and subtrochanteric fractures are often treated with internal fixation. However, the specific treatment should be based on the patient's own age, fracture type, preinjury activity, mental status, and other comprehensive factors to develop an appropriate treatment plan. Artificial hip arthroplasty began in the 1940s, and after nearly 70 years of development and improvement, it has become one of the most mature joint surgeries [6]. According to the mode of operation, artificial hip arthroplasty can be classified into artificial hemiarthroplasty (HA) and total hip arthroplasty (THA), which requires replacement of the femoral head and acetabulum; HA is artificial femoral head replacement, which only replaces the femoral head. Compared to THA, HA has less trauma, less bleeding, and low economic cost, so it is suitable for patients with older age, low life expectancy, and more basic diseases. Some studies have pointed out that the dislocation rate of HA is significantly lower compared to that of THA, and the risk of local fracture is lower, which can be adopted as the first choice for elderly patients with hip fracture [7]. Hip arthroplasty is one of the safe and reliable methods for the treatment of hip fractures in the elderly. It has the advantages of walking on the ground in the early stage, reducing complications, which can be adopted as the first choice for the treatment of hip fracture in patients over 80 years old [8].

In the face of the high prevalence rate of hip injury, ensuring the quality and safety of surgery, scientific perioperative management and actively promoting healthy behavior are the key to enhance the quality of medical service [9]. Therefore, in this study, the HAPA model is adopted to guide perioperative nursing of artificial hip replacement and to explore its application effect in clinical rehabilitation nursing of hip replacement from a novel point of view, so as to provide a new direction for the rapid rehabilitation of this kind of patients [10]. Meanwhile, it provides a reference basis for other researchers to apply this model.

The article "Effect of Rehabilitation Nursing under the Guidance of the Health Action Process Approach Model on Perioperative Nursing Effect of Artificial Hip Arthroplasty: Effect on Promoting Quality of Life and Postoperative Rehabilitation" was retracted in 2023. Reasons: unreliable results or conclusions; concerns about the data; concerns about the peer review; concerns about the citations.

## 2. Patients and Methods

### 2.1. General Information

A total of 200 patients with hip arthroplasty treated in our hospital from January 2019 to July 2021 were enrolled. The patients were randomly assigned into the control group and study group. The former received routine nursing, and the latter received rehabilitation nursing under the guidance of the HAPA model. In the control group, the age was 63-77 years old, with an average of 67.42 ± 3.55 years, including 56 males and 44 females, while in the study group, the age was 64-78 years old, with an average of 67.31 ± 3.33 years, including 51 males and 49 females. There was no statistical significance in the general data. This study was permitted by the Medical Ethics Association of our hospital, and all patients provided informed consent.

Inclusion criteria were as follows: (1) patients who underwent unilateral hip arthroplasty for the first time mainly including patients with FNF, intertrochanteric fracture, and osteonecrosis of the femoral head; (2) elderly patients aged from 60 to 80 years; (3) the patients having no vision, abnormal hearing, and communication disorder; and (4) patients who voluntarily participate in this study and agree and sign the informed consent form.

Exclusion criteria were as follows: (1) patients with old fractures; (2) patients with multiple injuries; (3) patients complicated with a malignant tumor; (4) patients having serious pathological changes of the heart, brain, liver, and other organs; (5) patients with severe cognitive impairment and disturbance of consciousness; and (6) mental disorders or abnormal noncooperation.

Shedding criteria were as follows: (1) those who dropped out in the middle of the research process; (2) those who have serious complications in the course of the study and are not suitable to continue, such as, joint dislocation, thromboembolism, and periprosthetic fracture; (3) those who were transferred to other departments during the period of sudden other diseases during hospitalization; and (4) follow-up failure.

### 2.2. Treatment Methods

The control group received routine nursing intervention and preoperative nursing: (1) admission evaluation: we evaluated patients' general admission data, specialist evaluation, and admission education; (2) psychological nursing: we publicized disease-related knowledge to patients, ask their psychological needs, and answer questions patiently; (3) life care: we assist patients in their daily activities to meet their basic needs; (4) pain nursing: we observe the location, nature, and scope of pain, timely grasp the degree of pain through a pain score, and guide patients to divert attention and listen to music and other relaxation techniques to relieve pain; if necessary, use analgesics for patients; (5) other: we strengthen preoperative examination and prepare for operation. Operation day nursing: (1) before operation: we instruct patients to wear hospital clothes, abstain from alcohol and food, wait for operation, randomly measure blood sugar in the morning of operation, prepare anesthetic bed, and hand over surgical drugs and case and image data; (2) operation: we prepare ECG monitor and oxygen device, measure vital signs, randomly measure patients' blood sugar after operation, and check patients' consciousness, skin, drainage tube, and wound. Postoperative nursing: (1) general nursing: we monitor patients' vital signs, blood oxygen saturation, consciousness, and urine volume and drainage; (2) specialist nursing: we guide the posture, abduction, and neutral position of the affected limbs and observe the abnormalities of wound dressing, drainage, limb sensation, peripheral circulation, exercise, and blood circulation; (3) dietary guidance: we give patients nutritional support with high protein, rich vitamins, and high calories; and (4) discharge guidance: we inform patients of the importance of rehabilitation exercise, administer medicine on time, and review regularly.

The article "Effect of Rehabilitation Nursing under the Guidance of the Health Action Process Approach Model on Perioperative Nursing Effect of Artificial Hip Arthroplasty: Effect on Promoting Quality of Life and Postoperative Rehabilitation" was retracted in 2023. Reasons: unreliable results or conclusions; concerns about the data; concerns about the peer review; concerns about the citations.

The study group received rehabilitation nursing under the guidance of the HAPA model, and the specific measures were as follows:

1. Motivation stage: this stage is mainly preoperative intervention, in which the researchers use health education brochures, pictures, PPT, video, and other forms of hip arthroplasty in our department to provide intervention to the patients. The main results are as follows. (1) The related knowledge of hip joint disease includes the anatomical structure, function, etiology, epidemiology, clinical characteristics, risk factors, and main manifestations of hip joint disease. (2) The early warning explanation of complications mainly includes lower limb venous thrombosis, stress injury, pulmonary infection, urinary system infection, incision infection, joint stiffness, joint dislocation, and prosthesis loosening. (3) The early warning explanation of adverse prognosis mainly includes dislocation of the hip joint, malnutrition, slow healing, joint contracture deformity, prolonged hospital stay, and increased economic burden. (4) The outline of the interview with the expected outcome of perioperative rehabilitation is as follows: what is your expectation of physical health? What are your expectations for this hospitalization? To what extent do you hope to achieve the rehabilitation effect after hip arthroplasty? According to the interview outline, make an appointment with the patients, conduct a face-to-face interview, introduce the purpose and content of the interview, use the Likert 5-level expected evaluation of the results (1 indicates no expectation, 2 indicates some expectation, 3 indicates general expectation, 4 indicates moderate expectation, and 5 indicates great expectation), record the questions or concerns raised by the patients in the interview, and edit and save the document. Targeted counseling was carried out on the problems existing in the patients in the interview. Communicate with team members about unanswered psychological or disease problems and solve them. (5) Explain the benefits of postoperative exercise training: pain relief, beneficial functional recovery, prevention or reduction of complications, early rehabilitation, shortening hospital stay, reducing economic burden, and returning to family and society more quickly. (6) The sharing of successful cases is as follows: the comparative display of the rehabilitation of the same patient before and after operation, the display of walking aids for patients with good rehabilitation, and so on. (7) To give social support, actively communicate with relatives to tell them to give psychological comfort and support to patients and give appropriate spiritual encouragement
2. Will decision stage: in the first part, formulate the rehabilitation action plan according to the *Practical Orthopaedic Rehabilitation Nursing Manual* edited by Ning Ning and Hou Xiaoling and the *Guide Manual of Perioperative Self-Rehabilitation Training for Patients*. The main results are as follows: (1) to formulate a rehabilitation exercise plan after artificial hip arthroplasty for functional training and rehabilitation guidance; (2) to formulate a self-care ability guidance plan for daily life, which can be used to guide life activities; and (3) to make a diary of rehabilitation exercise after artificial hip arthroplasty, which can be used to supervise patients and behavior regulation. In the second part, implement the rehabilitation action intervention and behavior regulation. (1) Every morning, members of the rehabilitation nursing team make joint rounds to understand and test the rehabilitation situation of the patients the day before and control the progress of rehabilitation. (2) Rehabilitation therapists conduct face-to-face and one-to-one bedside guidance on functional exercise according to the rehabilitation exercise plan after hip arthroplasty, until the patients fully learn and can repeat correctly. (3) In addition to routine nursing, the responsible nurses instructed the patients' daily activities according to the self-care ability guidance plan until the patients mastered various life skills and urged the patients to recover. (4) The researchers registered daily on the daily record sheet of rehabilitation exercise after artificial hip arthroplasty and recorded the basic information of patients and the time of operation on the day of operation. (5) The researchers guide the formulation and realization of the small and big goals of rehabilitation, such as ankle pump exercise 10 times a day, 4-6 groups per day. Instruct patients to give self-implied positive encouragement during daily exercise, such as I can and I believe I can do it. Ask the psychological status of the patients in the process of rehabilitation every day, and communicate with the psychological counselors to solve the unhealthy psychological problems and potential problems of the patients in time. (6) The WeChat communication group was established when the patients were discharged, and the patients or their family members could share the daily rehabilitation situation at any time. (7) After discharge, the patients were followed up by telephone once a week, and one month after operation, the patients were followed up and reexamined in the orthopaedic department of our hospital

The article "Effect of Rehabilitation Nursing under the Guidance of the Health Action Process Approach Model on Perioperative Nursing Effect of Artificial Hip Arthroplasty: Effect on Promoting Quality of Life and Postoperative Rehabilitation" was retracted in 2023. Reasons: unreliable results or conclusions; concerns about the data; concerns about the peer review; concerns about the citations.

### 2.3. Observation Index

#### 2.3.1. Satisfaction

After consulting the literature and experts' discussion, we designed patients' follow-up satisfaction, with a total of 10 items, and recorded patients' satisfaction with follow-up management mode, health education, medical and nursing service, and appointment registration process. It is assigned into four dimensions: very satisfied, satisfied, general, and dissatisfied. Satisfaction rate = very satisfaction rate + satisfaction rate + general rate.

#### 2.3.2. Visual Analog Pain Scale (VAS)

The scale consists of a straight line of 100 mm, from the beginning to the end and any part before it is expressed as the degree of pain of the patient. The beginning of the scale is 0 and the end of the scale is 100, which represents the degree of pain such as painless and unbearable, respectively. The closer the score is to the end, the stronger the degree of pain is. It is specifically classified as 1-30 mm, 40-60 mm, 70 mm, and 100 mm, respectively, indicating mild, moderate, and severe pain. It has strong practicability and guidance in clinic, and its use is simple, economical, and accurate. It is easy to be accepted by most patients and has been widely employed in clinic. See Figure 1 for details.

#### 2.3.3. Harris Hip Joint Function Score

The Harris hip function scale consists of four parts: pain, function, deformity, and range of activity, including 10 items, with a total score of 100. The higher the score, the better the function of the hip joint. After being tested, the scale has high reliability and validity, and its correctness, stability, and internal consistency are also high after retest. Cronbach's coefficient after Chinese translation is 0.811-0.904. At present, this scale has been widely employed to evaluate the function of the hip joint.

The article "Effect of Rehabilitation Nursing under the Guidance of the Health Action Process Approach Model on Perioperative Nursing Effect of Artificial Hip Arthroplasty: Effect on Promoting Quality of Life and Postoperative Rehabilitation" was retracted in 2023. Reasons: unreliable results or conclusions; concerns about the data; concerns about the peer review; concerns about the citations.

#### 2.3.4. Timed Up and Go Test (TUGT)

This test is a method to quantitatively evaluate the dynamic balance ability and functional walking ability of elderly patients. A standard armchair and a chronograph are required to carry out the experiment. The specific methods are as follows: the subjects leaned against the seat with both hands on the armrest of the seat, keeping both upper limbs relaxed, and the indicator issued a “start instruction” to ask the patient to stand up from the seat. Then, use the walker to walk forward 3 m with a clear mark or marker at 3 m, turn around after arrival, and then return to the seat to sit down again; the activity from the start instruction to the return to the seat is timed. Chinese scholars have tested the reliability and validity of the test, and its repeated test reliability in normal people and patients is 0.96-0.99 and 0.93-0.99, respectively.

#### 2.3.5. Modified Barthel Index (MBI)

The scale is improved by Shan on the basis of the Barthel Index (BI) in 1989. It is adopted to evaluate the self-care ability of patients' daily life (one of the most commonly used scales of ADL). The content of the scale remained unchanged on the basis of the original scale, and the evaluation items retained the original 10 items of BI, with a total score of 100. The grade of the scale was enhanced from four to five, that is, complete dependence, maximum help, moderate help, minimum help, and complete independence. The grading of MBI is more detailed compared to that of BI, and it is more sensitive and applicable to evaluate patients' self-care ability. The test-retest reliability is 0.880-0.992, and the internal consistency Cronbach's coefficient is 0.929.

#### 2.3.6. Quality of Life Scale

The quality of life scale consists of four subscales, including physical, psychological, social, and health self-awareness, with a total of 29 items. Cronbach's *α* coefficient of the scale is 0.79~0.91. The scale was scored by 1-5 grades. The lower the score, the higher the satisfaction.

### 2.4. Statistical Analysis

In this study, the data were input by using Excel, and the data were analyzed by using IBM SPSS 25.0 statistical software. Measurement data are expressed as mean ± standard deviation and analyzed by the t-test; enumeration data are expressed as percentage (%) and analyzed by the *χ*2 test. The data obeyed the homogeneity of variance of normal distribution, and two independent samples *t*-test and repeated measurement analysis of variance were performed. The data did not obey the homogeneity of variance of normal distribution, and the nonparametric Mann-Whitney *U* test was carried out. The Grade data were analyzed using the Wilcoxon test. *P* value less than 0.05 is considered statistically significant while *P* value less than 0.01 is viewed as highly statistically significant.

The article "Effect of Rehabilitation Nursing under the Guidance of the Health Action Process Approach Model on Perioperative Nursing Effect of Artificial Hip Arthroplasty: Effect on Promoting Quality of Life and Postoperative Rehabilitation" was retracted in 2023. Reasons: unreliable results or conclusions; concerns about the data; concerns about the peer review; concerns about the citations.

## 3. Results

### 3.1. Comparison of Nursing Satisfaction

First of all, we compared the nursing satisfaction: in the study group, 86 cases were very satisfied, 8 cases were satisfied, and 6 cases were general, and the satisfaction rate was 100.00%; in the control group, 48 cases were very satisfied, 22 cases were satisfied, 12 cases were general, and 18 cases were dissatisfied, and the satisfaction rate was 82.00%. Moreover, the nursing satisfaction in the study group was higher compared to that in the control group (*P* < 0.05). All the data results are indicated in Figure 2.

### 3.2. Pain Score Comparison

Secondly, we compared the pain scores. Before nursing, there exhibited no significant difference (*P* > 0.05). After nursing, the pain score of the two groups increased. Furthermore, the pain score of the study group at discharge and 1 month, 3 months, and 6 months after operation was lower compared to that of the control group (*P* < 0.01). All the data results are indicated in Table 1.

### 3.3. Comparison of the Harris Hip Joint Function Score

Thirdly, we compared the Harris hip function score. Before nursing, there exhibited no significant difference (*P* > 0.05). After nursing, the Harris hip function score of the two groups increased. And the Harris hip function score of the study group at discharge and 1 month, 3 months, and 6 months after operation was higher compared to that of the control group (*P* < 0.01). All the data results are indicated in Table 2.

### 3.4. Comparison of the Timed Stand-Up-Walking Test

Then, we compared the timed stand-up-walk test. Before nursing, there exhibited no significant difference (*P* > 0.05). After nursing, the time of the timed stand-up-walk test in both groups decreased. Of note, the timed stand-up-walk test at discharge and 1 month, 3 months, and 6 months after operation in the study group was lower compared to that in the control group (*P* < 0.01). All the data results are indicated in Table 3.

### 3.5. MBI Scoring Comparison

Next, we compared the MBI scores. Before nursing, there exhibited no significant difference (*P* > 0.05). After nursing, the MBI scores of the two groups increased. The MBI scores of the study group at discharge and 1 month, 3 months, and 6 months after operation were higher compared to those of the control group (*P* < 0.01). The results of all the data are indicated in Table 4.

The article "Effect of Rehabilitation Nursing under the Guidance of the Health Action Process Approach Model on Perioperative Nursing Effect of Artificial Hip Arthroplasty: Effect on Promoting Quality of Life and Postoperative Rehabilitation" was retracted in 2023. Reasons: unreliable results or conclusions; concerns about the data; concerns about the peer review; concerns about the citations.

### 3.6. Comparison of Quality of Life Scores

Finally, we compared the scores of quality of life. Before nursing, there exhibited no significant difference (*P* > 0.05). After nursing, the scores of quality of life decreased. And the scores of physiological function, psychological function, social function, and health self-cognition in the study group were lower compared to those in the control group (*P* < 0.01). All the data results are indicated in Table 5.

## 4. Discussion

The rapid development of population aging is a major population problem that cannot be ignored in China [11]. At present, people aged 60 or 65 and over are internationally defined as elderly people [12, 13]. China's aging has the characteristics of large proportion and rapid growth rate and will enter a high-speed aging development period from 2020 to 2030 [14–16]. The elderly group has the characteristics of aging of the body system, decline of function, and weakening of cognition with the increase in age, and the greater the physical, psychological, and social health problems, the greater the demand for social services [17, 18]. Some studies have predicted that the number of hip fractures in the United States will reach between 458000 and 1.037 million in 2050, and the number of cases in China will reach 1.079 million, with a high mortality rate of 8.9-13.9% within 30 days [18]. A large number of clinical practices have proved that this operation can effectively enhance the health-related quality of life of patients and significantly promote the quality of life. It is especially beneficial to the elderly [19]. Therefore, the demand for hip replacement is also growing in various countries. Some studies have estimated that the demand for the first total hip replacement in the United States will reach 57200 cases in 2030 [20]; in the United Kingdom, about 160000 people will receive joint replacement every year [21]. In China, the number of hip and knee replacements reached 951965 in 2019, with an annual growth rate of 38.25%, and hip prostheses accounted for 59.44% [22]. While the demand is increasing, it also brings a lot of pressure to the existing medical staff.

As a necessary condition for disease rehabilitation, rehabilitation nursing can assist and promote the overall physical, psychological, social, and mental health recovery of patients and plays an important role in the perioperative treatment of patients [23]. The study indicates that rehabilitation nursing is beneficial to facilitate patients' blood circulation, enhance muscle strength, prevent the risk of joint stiffness and dislocation, and effectively reduce pain and promote rehabilitation [24]. Scholars actively explore relevant measures to improve the rehabilitation care of patients undergoing hip replacement in order to promote their better recovery [23, 24]. In order to promote the transformation of individual behavior, a variety of health behavior theories are constantly innovating [25]. The more prominent one is a new social cognitive model created by a German psychologist in the 1990s: HAPA model. The model is a social cognitive model that effectively links intention and behavior, pays attention to the integrity of people in the environment, and can be employed to adopt, promote, and maintain each stage of the whole process of intervention behavior [26]. At present, the HAPA model has been widely used in various fields of society, but it is rarely used in my country. In studies in the field of orthopedics, the HAPA model has only achieved good results in the application of knee joint patients [27].

The article "Effect of Rehabilitation Nursing under the Guidance of the Health Action Process Approach Model on Perioperative Nursing Effect of Artificial Hip Arthroplasty: Effect on Promoting Quality of Life and Postoperative Rehabilitation" was retracted in 2023. Reasons: unreliable results or conclusions; concerns about the data; concerns about the peer review; concerns about the citations.

The HAPA model was first put forward by the German psychologist Ralf Schwarzer in 1992 [28]. This model draws lessons from Bandura's self-efficacy theory, integrates other models and theoretical contents related to health behavior and social cognition, and is a new social cognitive theoretical model to adopt, predict, and explain the process of health behavior and intervene to promote health behavior [29]. This model combines continuity and stage model and is a new orientation in the field of health behavior. The HAPA model integrates internal and external environmental factors that affect individuals and includes a variety of social cognitive variables for health behavior changes [30]. According to the HAPA model, the generation, maintenance, and recovery of healthy behavior are the result of the interaction of individual cognition, behavior, and emotion. Behavior change includes two stages: motivation and will determination [31]. In the motivation stage, generate behavioral intention, including risk perception, outcome expectation, and self-efficacy of the main cognitive predictive variables. The variables are defined as follows: risk perception refers to the understanding of the harm and severity of unhealthy behavior, result expectation is to predict the consequences of the behavior, and self-efficacy refers to the individual belief in the completion of an activity. Self-efficacy plays a dominant role in the model, followed by outcome expectation, and risk perception acts indirectly on behavior [31]. In the will determination stage, aim to convert intention into behavior and promote and maintain healthy behavior. This stage can be assigned into action plan, action, and behavior maintenance, including action plan, action control, and other variables [32]. The generation of intentional decision-making is a prerequisite for behavior, and planning is the intermediary of behavior change. The HAPA model explains the process of behavior change very well. According to the model, the individuals in each stage are defined as preintenders, intenders, and actors, and many scholars have paid attention to the HAPA model. It is found that some studies have widely employed the HAPA model to describe, explain, prevent, and intervene in various behaviors of individuals of different ages, such as diet and sleep health, vaccination, safe driving, skin protection, oral health, physical exercise, and sports injury prevention. Medical treatment is mainly employed in the study of disease rehabilitation behavior, patients' medication compliance, and physical activity [33]. Moreover, Chinese scholars pay attention to the application of the HAPA model which is relatively late. The HAPA model is mainly adopted in physical exercise, psychology, public health, health care, medical care, and other fields in China. The HAPA model has a good universality; the model is widely employed and achieved remarkable results, especially in the medical and health field, which provides a new perspective for the intervention of health behavior [34]. This study also has weaknesses including poor sample representation, erroneous control selection, and recall bias in exposure history. However, in order to obtain reliable results, we did our best to avoid them during the study.

The article "Effect of Rehabilitation Nursing under the Guidance of the Health Action Process Approach Model on Perioperative Nursing Effect of Artificial Hip Arthroplasty: Effect on Promoting Quality of Life and Postoperative Rehabilitation" was retracted in 2023. Reasons: unreliable results or conclusions; concerns about the data; concerns about the peer review; concerns about the citations.

Conclusively, the perioperative rehabilitation nursing program of artificial hip replacement for the elderly based on the HAPA model is feasible and effective, which can promote the functional recovery of hip joint, enhance the ability of self-care of daily life, relieve pain and anxiety, and help to achieve dynamic balance and gait stability in the early stage. The rehabilitation program is better than routine nursing. As a new social cognitive model, the HAPA model is applied to the rehabilitation nursing environment of hip replacement from the aspect of social cognitive behavior, which can help to change the rehabilitation behavior of elderly patients, playing an important role in the rehabilitation effect of perioperative nursing.

## Figures and Tables

**Figure 1:** VAS scoring.

**Figure 2:** Comparison of nursing satisfaction between the two groups.

**Table 1:** Comparison of pain scores between the two groups ($\bar{x}\pm s$, points).

Group	*N*	Before nursing	When discharged from the hospital	One month after operation	3 months after operation	6 months after operation
C group	100	7.43 ± 1.55	6.31 ± 0.22	5.33 ± 0.21	3.69 ± 0.52	1.56 ± 0.32
R group	100	7.49 ± 1.65	4.31 ± 0.31	3.19 ± 0.66	2.18 ± 0.21	0.55 ± 0.12
*t*		0.265	52.613	30.897	26.925	29.552
*P*		>0.05	<0.01	<0.01	<0.01	<0.01

**Table 2:** Comparison of the Harris hip joint function score between the two groups ($\bar{x}\pm s$, points).

Group	*N*	Before nursing	When discharged from the hospital	One month after operation	3 months after operation	6 months after operation
C group	100	56.22 ± 4.64	60.34 ± 3.42	68.66 ± 4.76	75.63 ± 3.53	80.23 ± 3.66
R group	100	56.65 ± 4.31	65.66 ± 3.66	78.34 ± 2.31	86.23 ± 3.77	90.52 ± 3.74
*t*		0.678	10.620	18.295	20.524	19.664
*P*		>0.05	<0.01	<0.01	<0.01	<0.01

**Table 3:** Comparison of the timed stand-up-walk test between the two groups of patients ($\bar{x}\pm s$).

Group	*N*	Before nursing	When discharged from the hospital	One month after operation	3 months after operation	6 months after operation
C group	100	53.98 ± 3.12	48.39 ± 4.21	34.69 ± 3.11	26.39 ± 1.25	14.82 ± 3.34
R group	100	53.59 ± 3.55	41.39 ± 3.31	28.49 ± 2.21	13.48 ± 1.35	5.68 ± 0.66
*t*		0.825	13.070	16.250	70.169	26.846
*P*		>0.05	<0.01	<0.01	<0.01	<0.01

**Table 4:** Comparison of the MBI score between the two groups ($\bar{x}\pm s$, points).

Group	*N*	Before nursing	When discharged from the hospital	One month after operation	3 months after operation	6 months after operation
C group	100	33.55 ± 3.41	46.42 ± 3.77	54.24 ± 5.67	78.77 ± 4.54	88.21 ± 3.66
R group	100	33.53 ± 3.67	58.13 ± 4.31	65.86 ± 3.53	84.64 ± 5.23	98.71 ± 4.63
*t*		0.039	20.449	13.397	8.475	17.790
*P*		>0.05	<0.01	<0.01	<0.01	<0.01

**Table 5:** Comparison of quality of life scores between the two groups before treatment ($\bar{x}\pm s$, points).

Group	*N*	Physiological function		Psychological function	Social function			Healthy self-cognition	
		Before nursing	After nursing	Before nursing	After nursing	Before nursing	After nursing	Before nursing	After nursing
C group	100	15.84 ± 4.91	13.86 ± 2.95	16.94 ± 3.91	14.85 ± 4.86	18.82 ± 3.95	16.37 ± 2.81	15.98 ± 3.91	13.86 ± 1.85
R group	100	15.96 ± 4.52	11.84 ± 2.91	16.95 ± 3.86	12.81 ± 1.85	18.84 ± 3.55	12.84 ± 3.81	15.87 ± 3.66	10.83 ± 2.91
*t*		0.179	4.874	0.018	3.922	0.037	7.456	0.205	8.787
*P*		>0.05	<0.01	>0.05	<0.01	>0.05	<0.01	>0.05	<0.01

## Data Availability

No data were used to support this study.
